# Analysis of Diabetes Disease Risk Prediction and Diabetes Medication Pattern Based on Data Mining

**DOI:** 10.1155/2022/2665339

**Published:** 2022-10-03

**Authors:** Lindong Zhang, Min Liu

**Affiliations:** The First School of Clinical Medical Sciences, Guangzhou University of Chinese Medicine, Guangzhou, Guangdong 510000, China

## Abstract

Diabetes mellitus is the second most common disease after cardiovascular diseases and malignant tumors. With the continuous acceleration of people's living standards and life rhythm, the number of diabetic patients is rapidly increasing and showing a trend of youthfulness. A recent study found that 114 million adults in China have diabetes and have a high prevalence rate, but the awareness rate, treatment rate, and compliance rate are low. If diabetes is not treated and controlled in time, various complications will occur, such as cardiovascular, cerebrovascular, and diabetic foot, which will not only have a great impact on the survival of the patient, but also cause a lot of pressure on the family and society. Therefore, prevention and control of diabetes is an important strategy to save medical resources and reduce medical costs. In this paper, we mainly read a lot of literature and accumulate some important theoretical knowledge to clarify the basic principles and methods of data mining and refer to the research results of other scholars to select a new combined algorithm model combining K-means algorithm and logistic regression algorithm to construct a prediction model of diabetes and explore the law of medication for diabetic patients based on this analysis.

## 1. Introduction

Diabetes mellitus (DM) is a metabolic abnormality syndrome caused by the interaction of genetic and environmental factors, mainly characterized by chronic hyperglycemia. As the standard of living of our people continues to improve, diabetes has had a significant impact on their quality of life, and its dangers have become a major public health issue. At the World Diabetes Conference 2015, the International Diabetes Federation recently published a report on diabetes, which mentioned that 415 million adults worldwide have diabetes, or 1 in 11. 110 million people in China have diabetes, the most common disease in the world [1]. Without intervention, the number of diabetics will increase geometrically by 2040. In the last 30 years, the prevalence of diabetes in China has increased from 0.67% to 11.6%. In Preventing Type 2 Diabetes in China (2013 Edition)3, it is stated that the main incidence group in China today is type 2 diabetes, 90% of which are middle-aged and elderly people. According to studies with relevant information, the prevalence of diabetes is more than 20% among patients aged 60 years and above. Its incidence is 10 times higher than that of the young population aged 20-30. Moderated by other factors, the incidence of diabetes rises by 68% for every 10 years of growth. The rapid increase in the incidence of diabetes in our country is mainly due to the following factors [2]. Firstly, changes in lifestyle. The decreasing availability of manual labour in society and the high utilisation of medical resources have led to an increasing incidence of diabetes. Secondly, changes in diet. As people's standard of living increases, the incidence of diabetes increases along with the prevalence of obesity. Thirdly, the ageing of the population and genetic factors etc. [3].

According to the latest data from the International Diabetes Federation, the worldwide prevalence of diabetes reached 8.3% in 2013 [4], and the number is growing rapidly [2]. It is estimated that by 2035, approximately 592 million people worldwide will have diabetes, and approximately 46% of these people will be undiagnosed. Data show that the number of deaths from diabetes complications worldwide is approximately 5.1 million, with medical costs of $548 billion, or 11% of total world health spending, and is projected to reach $627.3 billion in 2035. Currently, there are 114 million people with diabetes in the country, and 50.1% of them are “reservists” with diabetes. The potential incidence of diabetes is as high as 15.5%, and 60.7% of diabetic patients do not receive timely treatment and preventive education [5].

According to the China Statistical Yearbook, the share of health care in per capita consumption was 6.9% in 2013, an increase of 4.2% from 1990 [6]. This indicates that in addition to the rising cost of health care, the importance of health management is also increasing, which is an important reason for increasing health care spending. Health management is a subject of increasing interest in recent years, and its development will be more promising. Tertiary prevention is implemented to spread health knowledge and transform poor lifestyles in order to prevent and control risks [7].

At present, the prevention and treatment of diabetes in China has established the policy of “government-led, universal participation, prevention-oriented, combined with control, active initiation, and steady progress,” but the prevalence and mortality of diabetes are still high. The reason for this is that the early diagnosis and screening techniques for diabetes are not yet perfect [8], so many patients are already in the middle or late stage when they are diagnosed; in addition, the efficacy and prognosis of diabetes are very poor, and the domestic investment in primary and secondary prevention of diabetes is obviously insufficient, and there is also a lack of effective prevention and intervention means; finally, due to its complications, the quality of life of diabetic patients decreases [9], causing a great medical burden to families and society. Finally, due to its complications, the quality of life of diabetic patients decreases, causing a great medical burden to families and society. Therefore, risk prediction for diabetic patients can provide both early warning and comprehensive, continuous and proactive management to promote health and improve quality of life [10].

Most current healthcare information systems are limited to one-way data collection and statistics, lacking methods to summarize medical and health data, acquire knowledge and information, and proactively manage [11], feedback, and intervene on the information already available[5]. Data mining is an important technical tool that can extract the needed data from the massive amount of data. Therefore, the research in this thesis focuses on the use of various data mining techniques to develop diabetes risk prediction models and analyze their drug use patterns for the purpose of preventing and controlling the development of diabetes [12].

## 2. Introduction to Related Technologies

### 2.1. Data Mining Techniques

The concept of data mining was first introduced at the 11th International Joint Conference on Artificial Intelligence (IJCAI) in August 1989. Data mining is a technique to transform data into knowledge; it will collect data in a targeted way and analyze it and transform it into useful knowledge. Among these rules, data mining needs to follow the following rules:

1. The data mining target is large and high-dimensional data
2. The result of data mining is understandable and useful knowledge
3. Data mining is data-based and provides support for decision making

#### 2.1.1. Processes Underlying Data Mining

The usual data mining includes the following: target understanding, data collection, data pre-processing, model building, model evaluation, and execution [13]. The flow chart of data mining is shown in Figure 1.

1. Objective understanding. The initial work focuses on understanding the target needs of the project and translating the knowledge learned into data mining problems
2. Data acquisition. Based on this, the data objects to be performed are collected, and the required data are stored in a database or data warehouse [14]
3. Data preprocessing. This includes data integration, data attribution, data cleaning, and data conversion
4. Modeling. Depending on the data and mining objectives, appropriate analytical tools such as SPSS

Clementine, Wika, etc. are identified. Bayesian networks, association rules, decision trees, networks, cluster analysis and other relevant models can be built for the needs of data mining.

(5) Model evaluation. By comparing the existing accurate results or confirming them by experts
(6) Model implementation. The obtained knowledge is stored in a knowledge base for use by other applications

Data mining can be thought of as a cyclical process of operation, where if each step fails to achieve the goals set before mining, then you will go back to the previous step, make adjustments again, and execute again [15].

### 2.2. K-Means Algorithm

Clustering is the effective classification of similarities between different data items in a collection of data; each resulting set is called a cluster [16]. Clustering is an unsupervised learning method that provides only the attribute values of the data items without giving the classification values of the data items and its main goal is to put other types of data items into a cluster. The original data was analyzed and studied in depth using the clustering algorithm, and it was possible to discover the specific location of each data item and to compare the attributes in the dataset based on the experimental results [17].

The K-means algorithm is a typical distance-based clustering method, which uses distance as a measure of similarity, meaning that the shorter the given distance, the more similar it is.

The key to the K-means algorithm is to choose the *K*-value, which is an unsupervised learning algorithm that requires the experimenter to choose the *K*-value based on experience.

The algorithm proceeds as follows, and a simple diagram is shown in Figure 2.

1. Set *K* (assuming *K* = 2) as the initial cluster center of the algorithm, and choose *K* (assuming *K* = 2) arbitrarily in that original dataset
2. Compute each of the remaining data items separately, and classify them into clusters represented by the nearest centers according to the computed distances
3. Recalculate the centers of the clusters, and determine whether the centers have changed
4. Cycle 2-3 steps until the new cluster centers are equal to or less than the initial critical points, and the method is completed

### 2.3. Logistic Regression Algorithm

In the clinical application of diabetes, a dichotomous approach is generally used to classify the independent variables of patients into two categories [18]. Logistic regression algorithm models are divided into two types, quadratic and multiple, depending on the variable. The case of binary dependent variables is more common, that is, the output may have only two values, “0” and “1,” which represent meanings such as pass or fail, win or lose, live or die, and healthy or sick. Multiple logistic regression analysis occurs when there are more than two outcome types for the attribute values of a variable [19].

Logistic regression methods predict a finite number of dependent variables (two factors in Bernoulli's experiment) rather than a continuous one, compared to conventional linear regression methods. Moreover, linear regression is not meaningful for predicting binary variables. What we want to do is to transform the binary variables into variables that can withstand all the true values (positive or negative) [20]. To achieve this, binomial logistic regression first divides the probability of an event into individual independent variables at each level, scales them (continuously but not negatively), and establishes a continuous criterion for their logarithm (i.e., logit or log-odds) as a transformed version of the by variable.

The analytical study conducted in this thesis for diabetes focuses on a binary logistic regression algorithm model, which is based on a linear regression algorithm model of the following formula:

(1) $$\begin{array}{c} \text{P}=\alpha +\beta_{1}{\text{x}}_{1}+\beta_{2}{\text{x}}_{2}+\cdots +\beta_{\text{m}}{\text{x}}_{\text{m}}, \end{array}$$

where *m* is the number of independent variables.

The formula for the logistic regression algorithm model is defined as follows, where Figure 3 shows a simple example of the Sigmoid function transformation curve.

(2) $$\begin{array}{c} \mathrm{Pr}=\left\{\text{Y}=+1\left|{\text{X}}_{1},{\text{X}}_{2}\cdots {\text{X}}_{\text{d}}\right.\right\}=\sigma \left(\sum 1\leq \text{i}\leq \text{d}\beta_{\text{i}}{\text{X}}_{\text{i}}+\sum 1\leq \text{i}<\text{j}\leq \text{d}\beta_{\text{i},\text{j}}{\text{X}}_{\text{i}}{\text{X}}_{\text{j}}\right),\\ \mathrm{Pr}\left(\text{Y}=+1\left|\text{X}\right.\right)\sim \beta ∙\text{X},\\ \mathrm{Pr}\left(\text{Y}=-1\left|\text{X}\right.\right)=1-\mathrm{Pr}\left(\text{Y}=+1\left|\text{X}\right.\right),\\ \sigma \left(x\right)≔\frac{1}{1+e^{-x}}\in \left[0,1\right], \end{array}$$

where Sigmoid function transformation is shown in Figure 3.

(3) $$\begin{array}{c} \mathrm{Pr}\left(\text{Y}=+1\left|\text{X}\right.\right)\sim \sigma \left(\beta ∙\text{X}\right)\text{ andPr}\left(\text{Y}=-1\left|\text{X}\right.\right)=1-\mathrm{Pr}\left(\text{Y}=+1\left|\text{X}\right.\right). \end{array}$$

## 3. Application Method Design

### 3.1. Combined K-Means and Logistic Regression Algorithm Model

Data mining technology has a broad application prospect in the diagnosis of diabetic patients, whether it is classification, clustering, or association analysis, which can provide relevant research basis for diabetic patients [21]. The correct use of data mining techniques can uncover the hidden information from the massive data. In this paper, an improved method based on K-means and logistic regression has been used to predict the combination, and the corresponding model is given. Its model flow chart is shown in Figure 4.

The application of this combined K-means and logistic regression algorithm model consists of the following 7 steps:

1. A test based on information from the UCI to obtain possible factors for diabetes
2. Screening of certain inappropriate and inconsistent data in the data preprocessing stage
3. The original data with categorical markers were eliminated using the K-means clustering algorithm
4. Determining the ratio of the remaining data volume to the total original data, and using new seed values if the ratio is less than 75%
5. Using supervised logistic regression algorithm to classify the remaining data
6. Validated the test results by accuracy, safety, and specification
7. Compared with the existing model and proved that this model outperforms the existing model

### 3.2. Experimental Data Pre-Processing

Data preprocessing is a key part of data mining, because data mining is a data-driven experiment. From the analysis of data characteristics and systems in the previous section, we can see that complete, accurate, adequate, and valid data is the basis of data mining; otherwise, it will inevitably lead to the failure of data mining “rubbish in, rubbish out.”

The preprocessing of medical data for diabetic patients is similar to the preprocessing of centralized mining, but also has its own characteristics, and is generally divided into the following steps:

1. Data selection: Irrelevant and redundant information is eliminated. For example, some information of the patient that is not related to the changing pattern of the condition can be eliminated
2. Data removal: This mainly includes the following: excluding noise, excluding abnormal data, correcting inconsistent data, making up for missing data, removing missing data, deleting missing data, replacing missing values with constants, means, and predicted values. This step is an important part of the data preprocessing process, which will directly affect the modelling and analysis of data mining
3. Data transformation: It transforms the integrated data into a data format that meets the requirements of data mining, including data formatting and digitization of text data, etc.
4. Simplicity of data: If the data has too many attributes or variables, not only will it not be able to construct models effectively, but it will also generate noise, so it must be processed with simple data
5. Processing of anomalous data (outliers): Mathematical methods, anomaly detection, cluster analysis, and other algorithms are used to process anomalous data

### 3.3. Analysis of the Implementation Process of the Combined Model Algorithm

The original data that cannot be correctly clustered are first filtered using the improved K-means method [22], and the remaining optimized data are used as input for the next layer. Then, the logistic regression method is used to classify the remaining data, and the final conclusion is the classification effect of the whole model.

In the experiment of applying the method to Pima Indian Diabetes data, it was also necessary to optimize the quality of the raw data using data preprocessing techniques to improve the efficiency of data mining [23]. First, the definition of each attribute and its relationship with diabetes were compared in detail, and a conclusion was drawn that 0 indicates no pregnancy and 1 indicates pregnancy experience. This arithmetic process reduces the complexity of the information and increases the processing speed of arithmetic operations.

When collecting information, various records are often lost, and statistical items are not standardized. For example, the values of diastolic blood pressure, fat thickness, and serum insulin are not likely to be zero, which indicates that some of them are true. In order to reduce the impact of missing values and nonsense values on the prediction results, this paper uses the “ReplaceMissingValues” filtering method, which replaces all missing values with the most common method or average. Here, the 0 values in the previously processed pregnancy count items do not have to be replaced.

One of the biggest drawbacks of the K-means algorithm on the WEKA tool platform is that the initial seed values are generated randomly, so the experimenter must determine the initial seed values based on his or her own project experience. The initial seed value of the K-means algorithm often has a direct impact on the clustering effect of the experimental data. To prevent random errors in the initial seed values, a number of effective methods were used in the experiment. The first step is to record the resulting values and arrange them in order, where each value corresponds to a value called “within cluster sum of squared errors,” and the smaller the value, the better the clustering effect. The experiment recorded all 10,000 values of “within cluster sum of squared errors,” which corresponded to 1-10,000 subvalues. The obtained high quality primary seed values will be used in the next stage. The second part is that at the end of the K-means algorithm, a cycle must be added. The data that could not be correctly clustered were excluded from the experiment, and the following formula was used to find the scale values. If the ratio exceeds 75%, the next level will be performed using the correct grouped data. If not, this algorithm will exit the loop and reset a new seed value. If after 10,000 uses, or after 10 seconds of use, a suitable initial seed value has not been found and that value is greater than 75%, the largest initial seed value, and the corresponding seed value will be selected. Based on initial experience and preliminary judgments, the initial value of the seed selected for this test was 100.

In Table 1, the final cluster results of the above processing are shown, where 458 were clustered into cluster0 to represent negative items, while the other 310 were clustered into cluster 1 to represent positive items. By comparing the distribution of the 768 data items in the original dataset (500 negative and 268 positive), 179 incorrectly clustered and 589 correctly clustered examples were finally obtained, with the correct clustering examples accounting for 76.69% of the total initial dataset.

In this paper, the K- means clustering method is used to classify the data into positive and negative categories with an initial seed number of 100. By this method, the data with classification errors can be classified as noise, which results in more accurate data. The initial set of data had 500 negative and 268 positive numbers. Classifying them with the clustering algorithm yielded 458 negative and 310 positive messages, which means that there were 200 incorrectly clustered data. After eliminating these messages, the number of instances in the remaining dataset reached 568, and this part of the data occupied 74% of the total dataset.

In the secondary stage, the logistic regression algorithm was used for classification analysis. As with the independent variable information items in the original dataset, there were two categories of positive and negative classification result attributes. The logistic regression algorithm in which *Y* is whether the subject is diabetic or not and *X* is the value of the eight attributes of the original dataset. Each factor *X* is assigned a coefficient value, called *β*, which represents the weight. The data were effectively analyzed by a logistic regression algorithm to obtain the weights of the variables, and the magnitude of each weight indicates the difference between *X* and *Y*. After completing the algorithmic model, new data were entered and the results were predicted for both positive and negative outcomes.

## 4. Experimental Analysis of Application Practice

### 4.1. Experimental Environment Setup

The tool used in this paper is the WEKA Waikato Intelligent Analysis Environment (WEKA), which contains a large number of preprocessing, classification, clustering and related classical classification, clustering and correlation algorithms. The visualization interface developed using WEKA makes the experimental subject data available for quick and easy experimentation. At the same time, using the basic information provided by WEKA, one can quickly master the operation of the platform and use WEKA's interface files to easily complete one's own calculations. Its interface diagram is shown in Figure 5.

The WEKA platform combines a large number of core models and visualization tools to provide the experimenter with a convenient human-machine interface for a wide range of different data collection. The original version of WEKA consisted of a Tcl/Tk front-end model algorithm and Makefile system to run machine learning and data mining experiments. Nowadays, this fully Java-based version is widely used in many ways, especially in teaching and research. Its main advantages are as follows:

1. Freedom of access to this tool platform for all interested parties
2. Portability: The Java-based development tool platform can be easily ported on other platforms
3. Combination of most effective data preprocessing and data modelling techniques
4. Easy-to-use graphical user interface

### 4.2. Dataset Preparation

The first dataset used in this paper is from the Pima Indian Diabetes data in the UCI (UCI) machine learning database, with a total of 768 items. The 768 subjects are a general public in the state of Arizona, USA, and the National Institute of Diabetes and Kidney Diseases will conduct ongoing research on the population in this region. Each data item includes eight basic attributes, all of which are numeric in type, including the individual's basic health status and health care screening. For each attribute value, some examples of this dataset are shown in Table 2.

### 4.3. Analysis of Experimental Results for Diabetes Prediction

The improved K-means and logistic regression combined prediction model was proposed in the previous chapter, and after applying it to the dataset and conducting related experiments, it was finally concluded that the combined K-means and logistic regression prediction model is very good. The experimental results presented on the WEKA tool platform are shown in Figure 6.

Tested on a dataset, this paper presents an improved combined K-Min-Logistic regression forecasting model and compares its performance with other models.

The improved K-means and logistic regression methods were used to analyze the experimental data, and the corresponding experimental results were obtained, as shown in Tables 3 and 4. The Kappa statistic value was 0.752, which exceeded 0.75 indicating that the method had good similarity. The prediction accuracies were 0.916, 0.964, 0.964, 0.752, and 0.957, respectively. The results showed an accuracy of 90.7%. The analysis of the experimental data showed the validity of this method.

### 4.4. Experimental Analysis of Medication Use Patterns in Diabetic Patients

According to the modified K-means and logistic regression prediction model, the drug use pattern of diabetic patients was studied. The experimental results showed that there were 283 T2DM patients with 187 herbal medicines, with Salvia divinorum being the highest with 243 cases, accounting for 85.87%.

The analysis of the medication use in T2DM patients revealed 21 clinically significant drug combinations, including 10 types of Dan Shen, Xuan Shen, Cang Zhu, Ge Ge Ge, Bai Zhu, Huang Lian, Huang Qi, Sang Zhi, Gui Yao, and Lycium.

In particular, two drugs were identified in the trial, pioglitazone and chlorosulfopropylurea. To verify this conclusion, we reviewed a large amount of literature, and based on the available studies, pioglitazone was indeed a risk factor for increased hospitalization rates. As the combination of pioglitazone and chlorosulfopropurea has been associated with some adverse effects in diabetic patients, it can be assumed that the above effects of pioglitazone and chlorosulfopropurea may increase the risk of re-hospitalization in hospitalized patients.

Drug rule data mining trials not only consider single data, but also do not act as a vertical dataset and may contain incomplete data. For example, many of the underlying data items are ignored because they have small variance and missing values. Also, the information does not distinguish type 1 from type 2 diabetes, so the results of the above trial do not reflect the differences in medication use rules between the two. This trial represents an attempt to use data mining techniques in this area. Therefore, future studies should use the same approach to analyze this electronic medical record in Virginia to further test and improve the existing medication rules.

## 5. Conclusion

The rapid growth of medical data and the development of data mining techniques have made the effective use of medical data a focus of attention. This paper combines data mining models with medical data features to analyze the disease and drug use of diabetic patients in clinical data and proposes a set of reasonable and appropriate prediction models for the risk of diabetes in high-risk groups based on the experience of a large number of researchers. The model has been analyzed through the WEKA platform, and its predictive accuracy has been found to be significantly improved over previous studies. The Pima Indian Diabetes dataset used in this paper is the standard for many studies on diabetes-related data mining, and these data were compared with other researchers. The strengths and weaknesses of the trial data were preprocessed in detail to ensure that they were correct, reasonable, and standardized. Finally, after comparing the improved K-means and Logistic regression methods, which have a prediction accuracy of up to 95.42% and a conclusion of better results in terms of average prediction, the analysis of diabetes medication patterns can be carried out by keyword design during the model experiments, yielding the highest frequency of Danshen, occurrence.

## Figures and Tables

**Figure 1:** Flow chart of data mining.

**Figure 2:** Illustration of the K-means algorithm process.

**Figure 3:** Sigmoid function transformation curve.

**Figure 4:** Combination algorithm model flow chart.

**Figure 5:** WEKA experiment tool interface.

**Figure 6:** Graph of experimental results.

**Table 1:** Result of the 2-means cluster of the initial dataset.

Number	Label	Quantity
1	cluster 0	458
2	cluster 1	310

**Table 2:** Sample of Pima Indian Dataset.

Preg	Plas	Pres	Skin	Insu	Mass	Pedi	Age	Class
1	89	66	23	94	28.1	0.167	21	tested_negative
0	137	40	35	168	43.1	2.288	33	tested_positive
3	78	50	32	88	31	0.248	26	tested_positive
2	197	70	45	543	30.5	0.158	53	tested_positive
1	189	60	23	846	30.1	0.398	59	tested_positive
5	166	72	19	175	25.8	0.587	51	tested_positive
0	118	84	47	230	45.8	0.551	31	tested_positive
1	103	30	38	83	43.3	0.183	33	tested_negative
1	115	70	30	96	34.6	0.529	32	tested_positive
3	126	88	41	235	39.3	0.704	27	tested_negative

**Table 3:** Result of the new dataset.

Item	Value (%)
Prediction accuracy	90.7
Precision	91.6
Recall	96.4
MCC	75.2
ROC area	95.7
Kappa statistic	75.2

**Table 4:** Comparison of the experiment.

Algorithm	Accuracy rate (%)
Our model	90.7
Random forest	79
MLP	78
Bayes net	77
J48	72
Logistic	72

## Data Availability

The dataset used in this paper are available from the corresponding author upon request.
